# Edaravone Combined with Clopidogrel Is Beneficial to Improve Efficacy, Neurological Impairment, and Life Function in Acute Cerebral Infarction Patients

**DOI:** 10.1155/2021/8030521

**Published:** 2021-10-14

**Authors:** Liao Wu, Ying Sun, Guihua Ni, Bo Sun, Xiaoyu Ni, Shikun Cai

**Affiliations:** ^1^Department of Neurology, The Affiliated Huaian No.1 People's Hospital of Nanjing Medical University, Huaian, Jiangsu 223300, China; ^2^Department of Neonatal Pediatrics, The Affiliated Huaian No.1 People's Hospital of Nanjing Medical University, Huaian, Jiangsu 223300, China

## Abstract

**Objective:**

This research aimed at investigating the efficacy of edaravone combined with clopidogrel on acute cerebral infarction (ACI) and its influence on the neurological deficit and life function.

**Methods:**

Totally, 154 ACI cases were included and then divided into the control group (CG) (*n* = 71) and research group (RG) (*n* = 83) according to the treatment methods. Patients in the CG were treated with clopidogrel alone, and those in the RG were under edaravone-clopidogrel combination therapy. The efficacy, adverse reactions, NIHSS score, cerebral hemodynamic indexes, and Fugl-Meyer scale (FMA) and Barthel index (BI) of activities of daily living (ADL) scores were observed.

**Results:**

Compared with before treatment, the symptoms of both groups were improved after treatment: the NIHSS scores decreased, FMA and ADL scores increased, and cerebral hemodynamic indexes were improved. Compared with the CG, the efficacy and cerebral hemodynamic indexes of the RG were better, the adverse reactions were equivalent, the NIHSS score was lower, and the ADL and FMA scores were higher.

**Conclusion:**

Edaravone combined with clopidogrel can effectively treat ACI and improve the neurological deficit and life function of patients.

## 1. Introduction

Acute cerebral infarction (ACI) is an ischemic disease caused by cerebral vascular occlusion or stenosis, which can lead to brain injury and neurological deficit [1]. It has extremely high mortality, disability, and morbidity [2]. And it is the second most fatal disease in the world [3]. However, most can be prevented or treated by effective means [4–6]. Therefore, how to effectively prevent or treat this kind of disease is the key focus of current medical research.

The key to the treatment is to effectively improve cerebral vascular obstruction. Clopidogrel is a thienopyridine antiplatelet drug, which can inhibit platelet aggregation induced by ADP, thereby improving stroke, myocardial infarction, or other peripheral artery diseases [7]. For example, Fukuuchi et al. [8] thought that clopidogrel was the first choice for treating noncardiac embolic cerebral infarction. Li et al. [9] proposed that clopidogrel could improve the efficacy of aspirin in the treatment of ACI. Cerebral ischemia induces an increase in free radicals, which brings about ischemic brain damage such as edema and neuropathy [10]. At the moment, the treatment methods of neuroprotection for ACI are also facing a severe test [11]. Edaravone is an antioxidant, which can effectively eliminate fat- or water-soluble peroxy radicals, thereby inhibiting neuronal cell death and improving brain injury symptoms [10, 12]. Kobayashi et al. [13] claimed that edaravone could effectively improve the neurological function of ACI. Enomoto et al. [14] found that edaravone could effectively improve the efficacy of intravascular reperfusion and play a reliable neuroprotective role.

Based on the above, this study explored the efficacy of edaravone combined with clopidogrel in the treatment of ACI and its influence on neurological deficits and vital functions. It aims to provide scientific and reliable data for the combination of edaravone and clopidogrel. See the specific report below.

## 2. Methods

### 2.1. General Data

This research included 154 routine ACI cases and assigned them into CG (*n* = 71) and RG (*n* = 83) in view of the treatment methods. Patients in the CG were treated with clopidogrel alone, while those in the RG were under edaravone-clopidogrel combination therapy. In the CG, there were 49 males and 22 females with an average age of 55.61 ± 8.92 years, comprising 32 cases of basal ganglia infarction, 21 of cerebellar infarction, and 18 of brainstem infarction; the time from onset to consultation was 5.44 ± 2.98 days. In the RG, there were 57 males and 26 females with an average age of 56.78 ± 8.19 years, comprising 35 cases of basal ganglia infarction, 27 of cerebellar infarction, and 21 of brainstem infarction; the time from onset to consultation was 5.92 ± 2.83 days. In terms of gender, age, infarction site, time from onset to consultation, history of smoking, and excessive drinking, there was no statistical difference (*P* > 0.05) (Table 1).

### 2.2. Inclusion and Exclusion Criteria

In this research, 202 ACI patients diagnosed by magnetic resonance imaging (MRI) or X-ray computed tomography were recruited first, and then those with cerebral hemorrhage, coma, drug allergy, mental disorder, and other brain organ diseases were excluded. Finally, 154 patients were included. They were divided into CG (*n* = 71) and RG (*n* = 83) based on the treatment methods. Thereinto, the CG was treated with clopidogrel alone, and the RG was under edaravone-clopidogrel combination therapy (Figure 1). All subjects signed an informed consent form according to the Declaration of Helsinki. This research was approved by the hospital ethics committee.

### 2.3. Treatment Methods

After admission, all patients' blood pressure was regulated, and symptomatic supportive treatments such as dehydration, anticoagulation, and glucose control were given to them according to different clinical manifestations. On this basis, the RG was given edaravone (Sinopharm Group Guorui Pharmaceutical Co., Ltd., National Medicine Standard H20080056) 30 mg and normal saline (Beijing Tiantan Biological Products Co., Ltd., National Medicine Standard S10870001) 100 ml intravenous drip twice a day and clopidogrel (Sanofi (Hangzhou) Pharmaceutical Co., Ltd., National Medicine Standard J20180029) 75 mg orally once a day, while the CG was given clopidogrel 75 mg orally once a day. It was conducted continuously for 14 days.

### 2.4. Outcome Measures

The efficacy of the two groups was observed and counted after treatment [15]: according to NIHSS results, it is divided into four degrees: cure, remarkably effective, effective, and ineffective as follows: cure: the NIHSS score decreases by more than 90%, and clinical symptoms such as dizziness basically disappear; remarkably effective: the NIHSS score is reduced by 46%–90, and the clinical symptoms such as dizziness are obviously relieved; effective: the NIHSS score is reduced by 18%–45%, and clinical symptoms such as vertigo are slightly relieved; ineffective: the NIHSS score and clinical symptoms are not dramatically improved or even aggravated. Total effective rate = (cure + remarkably effective + effective)/total number.

The adverse reactions of both groups were observed and assessed during the treatment, including nausea, vomiting, and dizziness.

The neurological deficits of the two groups were observed and analyzed before and after treatment and evaluated by the National Institutes of Health Stroke Scale (NIHSS). The total score of the NIHSS is 0–42, and the higher the score, the more severe the nerve damage. At the same time, the cerebrovascular hemodynamic indicators were detected by the cerebrovascular hemodynamic monitor (CVHD-3000 type), including mean carotid blood flow (Qmean), mean blood flow velocity (Vmean), peripheral resistance, and characteristic impedance.

The life function of the two groups was evaluated after 2 days of treatment, and the Fugl-Meyer scale (FMA) and Barthel index (BI) of activities of daily living (ADL) were used to evaluate the patient's upper limb motor function and independent living activities. The former has a total score of 0–66, and the score is directly proportional to the upper limb motor function; the latter has a total score of 0–100, and the score is directly proportional to the patient's independent living activity ability.

### 2.5. Statistics and Analysis

SPSS 22.0 was applied to data statistical analysis. The measurement data were expressed by mean ± SD, and the count data were represented as *n* (%). Whether the data conform to normal distribution was verified by K-S test. For those conforming to the normal distribution, independent-sample *T*-test, paired-sample *T*-test, and chi-square test were employed for difference analysis. Taking 95% as its confidence interval, the difference was statistically marked when *P* < 0.05.

## 3. Results

### 3.1. Efficacy of Edaravone Combined with Clopidogrel on ACI

The efficacy of two groups of patients is counted in Table 2. In the CG, 17 cases were cured, 21 were remarkably effective, 18 were effective, 15 were ineffective, and the total effective rate was 78.87%. In the RG, 25 cases were cured, 27 were remarkably effective, 23 were effective, 8 were ineffective, and the total effective rate was 90.36%. The rate in the latter was statistically higher than that in the former (*χ*^2^ = 3.975, *P*=0.046).

### 3.2. Safety of Edaravone Combined with Clopidogrel on ACI

The adverse reactions of two groups of patients after treatment are counted in Table 3. There were 7 cases of adverse reactions in the CG, including 2 of nausea, 3 of vomiting, and 2 of dizziness; the total incidence was 9.86%. There were 5 cases of adverse reactions in the RG, including 1 of nausea, 1 of vomiting, and 3 of dizziness; the total incidence was 6.02%. There was no obvious difference between the two groups (*χ*^2^ = 0.783, *P*=0.376). The safety of the two treatment schemes was equal.

### 3.3. Effect of Edaravone Combined with Clopidogrel on Neurological Deficits in ACI

The degree of neurological impairment was evaluated by the National Institutes of Health Stroke Scale (NIHSS). The NIHSS score of the CG before treatment was 14.81 ± 1.58 scores, and the score after treatment was 8.24 ± 1.59 scores, with statistically marked difference (*P* < 0.001). In the RG, the NIHSS score was 14.82 ± 1.37 scores before treatment and 11.69 ± 1.02 scores after treatment, and there was an obvious difference between before and after treatment (*P* < 0.001). After treatment, the NIHSS in the RG was lower than that in the CG (*P* < 0.001) (Figure 2). Cerebral hemodynamic indexes were measured by the cerebrovascular hemodynamic monitor. Among them, the Qmean, Vmean, peripheral resistance, and characteristic impedance of the CG were (7.23 ± 2.01) cm^3^/s, (13.42 ± 2.23) cm/s, (78.67 ± 4.08) kPa·s/m, and (16.05 ± 2.74) kPa·s/m; those of the RG were (9.15 ± 2.12) cm^3^/s, (16.77 ± 2.86) cm/s, (93.87 ± 3.97) kPa·s/m, and (13.47 ± 2.96) kPa·s/m. The Qmean, Vmean, and peripheral resistance of the CG were lower than those of the RG (*P* < 0.001), while the characteristic impedance was higher (*P* < 0.001) (Figure 3).

### 3.4. Edaravone Combined with Clopidogrel Improves the Life Function of ACI

The life function of patients after treatment was assessed via FMA and ADL scores. The FMA and ADL scores of the CG were 17.88 ± 5.01 and 41.25 ± 6.14 scores before treatment and 22.46 ± 4.73 and 69.91 ± 6.73 scores after treatment. Those of the RG were 18.04 ± 4.94 and 40.74 ± 6.59 scores before treatment and 26.62 ± 4.85 and 69.91 ± 6.73 scores after treatment. After treatment, FMA and ADL scores increased in both CG and RG, and both FMA and ADL scores were higher in the RG than in the CG (*P* < 0.001). This manifests that edaravone combined with clopidogrel can better improve the life function of ACI patients (Figure 4).

## 4. Discussion

ACI not only leads to the lack of energy and nutrients (such as sugar and oxygen) for maintaining the normal function of brain tissue but also causes metabolic dysfunction [16]. If patients cannot be treated promptly and effectively, recurrent stroke or cardiovascular adverse events may increase. Meanwhile, it has a great influence on neurological function, and improper treatment may affect its normal operation. Thus, finding an effective and reliable scheme to improve ACI and neurological function is urgent.

In this research, the efficacy of edaravone combined with clopidogrel is better than that of clopidogrel alone, which shows that edaravone does not affect the antiplatelet effect of clopidogrel, but promotes it. Simultaneously, the results of cerebral hemodynamics revealed that edaravone combined with clopidogrel was more beneficial to the recovery and improvement of vascular function. The neuroprotective effect of edaravone also effectively improved the neurological deficit caused by ACI. Follow-up results manifest that edaravone combined with clopidogrel can effectively promote the recovery of patients' daily life function.

Analyzing the reasons for the above results, clopidogrel is the second generation of thiophene-pyridine, which has good antiplatelet effect and can reduce the risk of recurrent ischemia time [17, 18]. Many studies have confirmed the outstanding performance of clopidogrel in ACI. For instance, Wang et al. [19] found that clopidogrel could effectively improve the prognosis of ACI treated with aspirin alone and reduce the risk of secondary stroke. Similarly, another research study [20] also showed that the use of clopidogrel could reduce the possibility of secondary stroke in the first 90 days. Edaravone is a powerful antioxidant, which is mainly used to treat acute ischemic events [21]. Kamouchi et al. [22] found that edaravone could effectively reduce the risk of acute kidney injury secondary to ACI. Edaravone is a potential neurovascular protective agent [23]. Wu et al. [24] confirmed that edaravone could eliminate OH−, NO, and ONOO− produced by ischemic stroke in a dose-dependent manner, thus inhibiting neuroinflammation.

However, due to time limit, this research still has some shortcomings, mainly as follows: first, this research did not track the long-term effects of the two treatment options on ACI; second, although this research considered that edaravone combined with clopidogrel had good efficacy and neuroprotective effect, it did not design further basic experiments to explore the specific mechanism. Hence, in subsequent studies, relevant *in vitro* or *in vivo* experiments should be designed to explore the main regulatory mechanisms of edaravone combined with clopidogrel in ACI. Third, more samples were not included in this research, and more subjects should be recruited in future studies.

To sum up, after comparing the efficacy and safety of clopidogrel monotherapy and edaravone-clopidogrel combination therapy in ACI, this paper holds that the safety of edaravone combined with clopidogrel is equivalent to clopidogrel monotherapy, but the efficacy is better. Edaravone combined with clopidogrel is more conducive to the recovery and improvement of neurological function and life function of patients. Hence, the combination therapy is worth to be popularized and applied.

## Figures and Tables

**Figure 1:** Flowchart.

**Figure 2:** Comparison of the NIHSS score (mean ± SD, scores). Note: compared with the same group before treatment, ^*∗*^*P* < 0.001; compared with the CG after treatment, ^#^*P* < 0.001.

**Figure 3:** Comparison of cerebral hemodynamic indexes (mean ± SD). Note: compared with the CG, ^*∗*^*P* < 0.001.

**Figure 4:** Comparison of the life function score (mean ± SD, scores). Note: compared with the same group before treatment, ^*∗*^*P* < 0.001; compared with the CG after treatment, ^#^*P* < 0.001.

**Table 1:** Comparison of general data.

Information	CG (*n* = 71)	RG (*n* = 83)	*t*/*χ*^2^	*P* value

Gender			0.002	0.964
Male	49	57		
Female	22	26		
Age (years)	55.61 ± 8.92	56.78 ± 8.19	0.848	0.398
Infarction site			0.181	0.913
Basal ganglia region	32	35		
Cerebellum	21	27		
Brainstem	18	21		
Time from onset to consultation	5.44 ± 2.98	5.92 ± 2.83	1.024	0.308
Hypertension			0.068	0.794
Yes	37	45		
No	34	38		
Diabetes			2.046	0.153
Yes	32	47		
No	39	36		
Hyperlipidemia			1.074	0.300
Yes	35	34		
No	36	49		
History of smoking			0.210	0.647
Yes	24	31		
No	47	52		
History of excessive drinking			0.008	0.931
Yes	33	38		
No	38	45		

**Table 2:** Comparison of efficacy (*n* (%)).

Group	Cure	Remarkably effective	Effective	Ineffective	Total effective rate

CG (*n* = 71)	17 (23.94)	21 (29.58)	18 (25.35)	15 (21.13)	56 (78.87)
RG (*n* = 83)	25 (30.12)	27 (32.53)	23 (27.21)	8 (9.64)	75 (90.36)
*χ* ^2^					3.975
*P* value					0.046

**Table 3:** Comparison of adverse reactions (*n* (%)).

Group	Nausea	Vomiting	Dizziness	Total incidence

CG (*n* = 71)	2 (2.82)	3 (4.23)	2 (2.82)	7 (9.86)
RG (*n* = 83)	1 (1.20)	1 (1.20)	3 (3.61)	5 (6.02)
*χ* ^2^				0.783
*P* value				0.376

## Data Availability

The data used during the current study are available from the corresponding author upon request.
